# Tibial nerve stimulation to inhibit the micturition reflex by an implantable wireless driver microstimulator in cats

This article has been retracted.

**DOI:** 10.1097/MD.0000000000004537

**Published:** 2016-08-19

**Authors:** Xing Li, Li-Min Liao, Guo-Qing Chen, Zhao-Xia Wang, Tian-Ji Lu, Han Deng, Gerald-E Loeb

**Affiliations:** a Rehabilitation School of Capital Medical University, Department of Urology at China Rehabilitation Research Centre; b Beijing Key Laboratory of Neural Injury and Rehabilitation; c Center of Neural Injury and Repair, Beijing Institute for Brain Disorders, Beijing, China; d University of Southern California, Los Angeles, USA.

**Keywords:** cat, implantable, microstimulator, micturition reflex, tibial nerve stimulation

## Abstract

**Background:**

Traditional tibial nerve stimulation (TNS) has been used to treat overactive bladder syndrome (OAB), but there are some shortcomings. Thus, a novel alternative is needed for the treatment of OAB. The study investigated the effects of a new type of tibial nerve microstimulator on the micturition reflex in cats.

**Methods:**

An implantable wireless driver microstimulator was implanted around the tibial nerve in 9 α-chloralose anesthetized cats. Cystometry was performed by infusing 0.9% normal saline (NS) or 0.25% acetic acid (AA) through a urethral catheter. Multiple cystometrograms were performed before, during, and after TNS to determine the inhibitory effect of the microstimulator on the micturition reflex.

**Results:**

TNS at 2 threshold (T) intensity significantly increased the bladder capacity (BC) during NS infusion. Bladder overactivity was irritated by the intravesical infusion of 0.25% AA, which significantly reduced the BC compared with the NS infusion. TNS at 2 T intensity suppressed AA-induced bladder overactivity and significantly increased the BC compared with the AA control.

**Conclusion:**

The implantable wireless driver tibial nerve microstimulator appears to be effective in inhibiting the micturition reflex during physiologic and pathologic conditions. The implantable wireless driver tibial nerve microstimulator could be used to treat OAB.

## 1 Introduction

Overactive bladder syndrome (OAB) is defined by the International Continence Society as “urgency, with or without urge incontinence, usually with frequency and nocturia in the absence of proven infection or other obvious pathology.”^[1]^ The prevalence of OAB in adult ranges from 10.2% to 17.4% in males and 7.7% to 31.3% in females.^[2]^ OAB is a common urologic disorder which seriously impacts the quality of life and imposes a substantial economic burden on the healthcare system.

Tibial nerve stimulation (TNS) has been verified as a minimally invasive treatment option for patients with OAB, and is recommended by a recent update of the AUA/SUFU guidelines for the management of OAB in adults as third-line treatment, as well as botulinum toxin A and sacral neuromodulation, in patients refractory to treatment with conservative strategies and pharmacologic therapy.^[3]^ Previous studies showed that the OAB animal model with cats could be induced by 0.25% acetic acid (AA) irritation. Following AA irritation bladder, C-fiber afferents were activated and OAB was induced including a marked reduction in bladder capacity (BC).^[4,5]^ The purpose of the present study was to determine the effects of acute TNS delivered by an implantable wireless driver microstimulator (NuStim device; GenralStim Inc., Hangzhou, Zhejiang, China) on the micturition reflex in normal and OAB cats.

## 2 Methods

### 2.1 Device introduction

The NuStim device consists of 3 subsystems (the stimulator, the radiofrequency [RF] cushion, and the android pad; Fig. 1). The stimulator has a cylindrical shape with 2 leads on each side (3 mm in diameter × 10 mm in length; Fig. 2). The stimulator receives RF electromagnetic pulses from an external machine, the RF cushion (Fig. 3), and transforms the RF electromagnetic pulses into current pulses. The stimulation parameters are as follows: 0 to 15 V, 2 to 20 Hz pulse rate, and 200 ms pulse width. The stimulation parameters can be adjusted immediately during the treatment using a remote control (an app from an android pad). The current pulse generated by the stimulator is a biphasic, asymmetric exponential pulse.

**Figure 1:** The schematic diagram of the NuStim device. RF = radiofrequency.

**Figure 2:** The stimulator: NuStim device.

**Figure 3:** The RF cushion: the RF cushion can receives bluetooth signal from the pad and generates RF signal to activate the stimulator. It is also the energy supply for the stimulator. RF = radiofrequency.

### 2.2 Experimental setup

Experiments were conducted in 9 cats (5 males and 4 females, 2.5–3.5 kg, 6–12 months old, domestic shorthairs) under α-chloralose anesthesia (65 mg/kg intravenously) after induction with isoflurane (2%–3% in oxygen). A tube was inserted to maintain airway access after a tracheotomy. Heart rate, blood oxygen level, and systemic blood pressure were monitored throughout the experiment. Fluid was administered via the cephalic vein. Body temperature was maintained with a heating pad. The Animal Care and Use Committee at the Capital Medical University approved all protocols involving the use of animals in this study (AEEI-2016-041).

Cats underwent implantation in the supine position after disinfection of the right hindlimb. A 2- to 3-cm incision was made on the medial side of the hindlimb above the ankle. The tibial nerve was exposed. Then, the stimulator was placed near the neurovascular bundle parallel to the tibial nerve and its cathode perpendicular to the cushion. During the procedure, the stimulator was activated to confirm function and placement. Toe movement was observed when the stimulator was properly positioned. The stimulator was fixed by a ligature around the neurovascular bundle if proper placement was confirmed and the wound was closed.

The ureters were isolated via an abdominal incision. The ureters were cut and drained externally. The bladder was inserted via a double lumen catheter through the urethra. The catheter was then secured by a ligature around the urethra. One lumen of the catheter was used to infuse the bladder with either 0.9% normal saline (NS) or 0.25% AA at a rate of 1 to 2 mL/min after connecting to a pump. The other lumen was connected to a pressure transducer to measure the bladder pressure. After completing the preparation work, stimulation was applied.

### 2.3 Stimulation protocol

Biphasic exponential pulses (200-μs pulse width, 6-Hz frequency) were delivered to the tibial nerve. By gradually increasing the stimulation intensity, the intensity threshold (T) inducing toe movement was determined. The BC was used to test the inhibitory effect of the stimulator. After the appearance of the first large-amplitude (>30 cmH_2_O) bladder contraction, the bladder infusion with NS or AA was stopped.^[4,5]^ First, after emptying the bladder, 2 or 3 cystometrograms (CMGs) with NS were performed without stimulation to obtain the control BC and assess the reproducibility. After the BC was stabilized, TNS (frequency, 6 Hz; intensity, 1–2 T) was applied during 2 sequential CMGs. Another CMG without stimulation was performed in the end. Second, after emptying the bladder, 0.25% AA was infused into the bladder to irritate and induce bladder overactivity during 3 to 5 CMGs (1 hour). After the BC stabilized, TNS (frequency, 6 Hz; intensity, 1–2 T) was applied again during 2 sequential CMGs. Another CMG without stimulation was performed in the end. The bladder was emptied after each CMG, and a 10-minute rest period was permitted between successive CMGs to allow the distended bladder to recover.

### 2.4 Statistical analysis

The Statistical Package for the Social Sciences (SPSS) version 19.0 (SPSS Inc., Chicago, IL) was used for statistical analysis. The level of significance was 0.05. To compare the repeated CMG recordings, the BCs were normalized to the measurement of the first control CMG during the NS or AA infusion. Repeated measurements of the same animal under the same CMG conditions were averaged. All summary data are expressed as the mean ± Standard error (SE). Statistical significance was detected by one-way Analysis of Variance (ANOVA) followed by Bonferroni posttests or Kruskal–Wallis test followed by Tamhane posttests.

## 3 Results

All of the cats were implanted successfully. There was no obvious bleeding or edema observed during the surgical procedure and stimulation process.

During infusion with NS, the large-amplitude (>30 cmH_2_O) and long-duration (>20 seconds) bladder contractions were induced when the BC reached the micturition volume (the first traces in Figs. 4 and 5). Compared with the baseline level (103.3 ± 8.5 mL), TNS at 1 T intensity did not significantly increase the BC (109.0 ± 19.7 mL; *P* = 1.00). TNS at 2 T intensity significantly increased the BC (147.1 ± 29.1 mL) compared to the baseline level (*P* = 0.03; Fig. 4). Irritation of the bladder with 0.25% AA-induced bladder overactivity and significantly reduced the BC (54.9 ± 18.4 mL) compared to NS infusion (*P* < 0.001). When TNS was applied at 1 T intensity, AA-induced bladder overactivity was not suppressed nor was the BC significantly increased (66.5 ± 20.1 mL; *P* = 0.22) compared to the AA control level. TNS at 2 T intensity suppressed AA-induced bladder overactivity and significantly increased BC (87.0 ± 28.1 mL) compared to the AA control (*P* = 0.01); the BC did not return to the NS control level (*P* = 0.88; Fig. 5). During the experiment, the CMGs were stable because the BC returned to the initial level after infusion of NS and AA when the stimulation was stopped (the fourth and fifth traces in Figs. 4 and 5).

**Figure 4:** TNS at 2 T intensity inhibits reflex bladder activity induced by intravesical infusion of 0.9% NS and significantly increases BC. Stimulation: pulse width 200 μs, frequency 6 Hz, intensity 1 V (2 T). Infusion rate: 1 mL/min. BC = bladder capacity, NS = normal saline, T = threshold, TNS = tibial nerve stimulation.

**Figure 5:** TNS at 2 T intensity suppresses bladder overactivity induced by intravesical infusion of 0.25% AA and significantly increases BC. Stimulation: pulse width 200 μs, frequency 6 Hz, intensity 1 V (2 T). Infusion rate: 1 mL/min. AA = acetic acid, BC = bladder capacity, T = threshold, TNS = tibial nerve stimulation.

## 4 Discussion

The tibial nerve is a mixed sensory and motor nerve containing L4-S3 fibers that originate from the same spinal segments as the innervations to the bladder and pelvic floor. The ankle region of TNS is close to the Sanyinjiao used in Chinese acupuncture.^[6]^ The technique has been used to treat lower urinary tract dysfunction, such as urgency, frequency, enuresis, incontinence, and retention of urine.^[7]^ Although the mechanism underlying TNS is not clear, a number of studies have been conducted to prove the efficacy of TNS in treating patients with OAB, especially for patients who are refractory to conservative treatments or experience intolerable side effects of drug therapy.^[8,9]^

Urgent® PC (Uroplasty Ltd., Manchester, UK) is an FDA-approved, minimally invasive, office-based neuromodulation system designed to deliver retrograde stimulation to the sacral nerve plexus through percutaneous electrical stimulation of the posterior tibial nerve.^[10]^ Urgent PC has been shown to be safe with statistically significant improvements in patient assessment of OAB, and with objective efficacy comparable to pharmacotherapy.^[11]^ However, the patients need a temporary insertion of a 34 gauge needle electrode, slightly cephalad to the medial malleolus each time, which may lead to bleeding, pain, and uncomfortable feelings. The procedure must be performed by a professional.

To overcome the disadvantage of Urgent PC, adhesive skin surface electrodes have been used instead of needle electrodes to treat OAB.^[12,13]^ Although adhesive skin surface electrode therapy is noninvasive and easily managed by patients, it may be less effective than percutaneous TNS, in part because of the indirect nerve stimulation.^[14]^ In addition, adhesive skin surface electrode therapy also needs a medical professional to identify the proper position of the surface electrode, just as for needle electrodes.

In 2006, a study reported an implant-driven TNS device (Urgent-SQ; CystoMedix Inc., Anoka, MN) in the treatment of refractory OAB.^[15]^ The device consists of an external electromagnetic pulse generator with RF transmission capability and an internal electromagnetic pulse receiver. Urgent-SQ has a similar working principle as the device used in this study; however, the external stimulator has to be placed directly on the skin with a cuff around the medial malleolus to activate the internal body and the implant is relatively long (approximately 4 cm). The implantation requires a 5- to 7-cm incision approximately 5 cm above the medial malleolus and parallel to the tibia under spinal or general anesthesia. Thus, this technique has not been widely used.

In this study, we performed the TNS procedure with an implantable wireless driver microstimulator (NuStim). NuStim consists of 3 subsystems (the implantable microstimulator, the RF cushion, and the android pad). The stimulator receives RF electromagnetic pulses from the RF cushion and transforms the RF electromagnetic pulses into current pulses. The stimulation parameters can be adjusted by a remote control (an app from an android pad). Even though we also implanted the stimulator via an open surgical procedure in this study, it can be performed in a fully percutaneous and simplified way in patients in the future as the implantation for the tined lead in the InterStim Therapy procedure (Medtronic, Minneapolis, Minn, US) because this microstimulator is only 3 mm in diameter and 10 mm in length (Fig. 2). The insertion surgical kit has now been produced and will be used for clinical trials. The other advantage of our microstimulator is that it does not require an integrated battery. The microstimulator receives RF electromagnetic pulses from the RF cushion and transforms the RF electromagnetic pulses into current pulses. Thus, the patients do not need to replace the stimulator when the battery is depleted, as with the InterStim.

In this study, we investigated the effects of acute TNS delivered by a microstimulator on the micturition reflex in normal and OAB cats, which revealed that TNS with the NuStim device implanted in the tibial nerve in cats is effective in not only inhibiting reflex bladder activity induced by intravesical infusion of NS, but also suppressing bladder overactivity induced by intravesical infusion of AA. TNS at 2 T intensity significantly increased BC compared to the baseline level during NS infusion (*P* = 0.03; Fig. 4) while suppressing AA-induced bladder overactivity and significantly increasing BC compared to the AA control (*P* = 0.01; Fig. 5). Our study showed similar results performed by direct TNS via the cuff electrode in cats^[4,5]^ and appears to be practical in treating patients with OAB via the implanted stimulator in the future.

OAB treatment needs repeated stimulation sessions long term or lifelong. This limits the use of traditional TNS. With the production of an insertion kit and wearable external electromagnetic pulse generator, the NuStim device is a minimally invasive neuromodulation technique for OAB patients. The NuStim is placed closer to the tibial nerve, which could produce a more effective stimulation. Patients can do activities, such as reading and watching TV, during the treatment. As a self-administered therapy without professional supervision, it can be easily taught to patients or their families and could be applied at home; however, we only investigated the acute effect of the NuStim device in this study and there was a lack of information on long-term therapy. Moreover, although there were no obvious side effects (i.e., bleeding or edema) in this study, it was still unknown whether it could induce pain, infection, and other complications or not. In addition, the biocompatibility of the implants needed to be determined during chronic use.

In conclusion, this study has demonstrated that TNS by an implantable wireless driver microstimulator (NuStim) is effective in inhibiting the micturition reflex during physiologic and pathologic conditions. Moreover, improved BC, which was observed in this study, is an encouraging finding that can be used as a potential treatment modality in the clinical practice of overactive bladder.

## Acknowledgments

The authors would like to thank the Natural Science Foundation of China and Beijing Natural Science Foundation for financially supporting this research. They also would like to thank Fangping Li, Fangxi Li, and Xue-Chen Huang for the supports for this study and the valuable discussion and suggestions.
